The article "Synthesis, Characterization, and In Vivo Cytokinome Profile of IL-12-Loaded PLGA Nanospheres" was published in 2022. Journal: J Immunol Res.

# Synthesis, Characterization, and *In Vivo* Cytokinome Profile of IL-12-Loaded PLGA Nanospheres

**DOI:** 10.1155/2022/6993187

**Published:** 2022-04-14

**Authors:** Ryan A. Lacinski, Justin E. Markel, Jabeen Noore, Hillary G. Pratt, Brock A. Lindsey

**Affiliations:** ^1^Department of Orthopaedics, West Virginia University, Morgantown, WV, USA; ^2^Department of Surgery, West Virginia University, Morgantown, WV, USA

## Abstract

We report the successful encapsulation and elution of recombinant murine IL-12 (rmIL-12) from poly(lactide-co-glycolic) acid (PLGA) nanospheres (IL-12-NS) synthesized using the double emulsion/solvent evaporation (DESE) technique with microsphere depletion through ultracentrifugation. Images obtained with scanning electron microscopy (SEM) showcased a characteristic spherical shape with a mean particle diameter of 138.1 ± 10.8 nm and zeta potential of −15.1 ± 1.249 mV. These values suggest minimal flocculation when in solution, which was reflected in an *in vivo* biodistribution study that reported no observed morbidity/mortality. Encapsulation efficiency (EE) was determined to be 0.101 ± 0.009% with average particle concentration obtained per batch of 1.66 × 10^9^ ± 4.45 × 10^8^ particles/mL. Disparate zeta (*ζ*) potentials obtained from both protein-loaded and protein-unloaded batches suggested surface adsorption of protein, and confocal microscopy of BSA-FITC-loaded nanospheres confirmed the presence of protein within the polymeric shell. Furthermore, elution of rmIL-12 from IL-12-NS at a concentration of 500 million particles/mL was characterized using enzyme-linked immunosorbent assay (ELISA). When IL-12-NS was administered *in vivo* to female BALB/c mice through retroorbital injection, IL-12-NS produced a favorable systemic cytokine profile for tumoricidal activity within the peripheral blood. Whereas IFN-*γ* nadir occurred at 72 hours, levels recovered quickly and displayed positive correlations postburst out to 25 days postinjection. IL-12-NS administration induced proinflammatory changes while prompting minimal counterregulatory increases in anti-inflammatory IL-10 and IL-4 cytokine levels. Further, while IL-6 levels increased to 30 folds of the baseline during the burst phase, they normalized by 72 hours and trended negatively throughout the sill phase. Similar trends were observed with IL-1*β* and CXCL-1, suggesting a decreased likelihood of progression to a systemic inflammatory response syndrome-like state. As IL-12-NS delivers logarithmically lower amounts of IL-12 than previously administered during human clinical trials, our data reflect the importance of IL-12-NS which safely create a systemic immunostimulatory environment.

## 1. Introduction

Immunostimulation is a rapidly evolving concept in the field of immunooncology. While once a controversial topic, it is now well-established that intact immune systems can kill tumor cells [1]. The indiscriminate cytotoxicity of innate immunity combined with the antigen-specific cell surface receptor repertoire of adaptive immunity forms a highly effective network of host defense mechanisms that manage bodily insults of various etiologies, including tumorigenic cell transformation [2–4]. Currently, the most successful application of tumor immunotherapy has occurred using anticytotoxic T-lymphocyte-associated protein 4- (CTLA-4-) and/or antiprogrammed death-ligand 1- (PD-L1-) directed monoclonal antibodies as adjuvant treatment for lung and skin cancers [5]. However, checkpoint blockade alone has repeatedly failed to improve survival in other cancers including metastatic sarcoma over the current standard of care [6], likely due to a combination of tumor-induced immunosuppressive forces that circumnavigate checkpoint blockade alongside extensive tumor cell pleomorphism [7]. Our group has shown that treatment modalities employing these “blocking the block” strategies can fail by prompting the emergence of tumor escape mechanisms [8].

Preclinical studies have shown that interleukin- (IL-) 12, an immunostimulatory cytokine, can induce strong antitumor responses against various malignancies. Compared to the monoclonal antibody checkpoint blockade, IL-12 is active over a broader spectrum of immune functions; examples of the effects of IL-12 include differentiation of T helper cells into the type one (T_H_1) phenotype, stimulation of interferon-gamma production by macrophages, and enhanced cytotoxicity of natural killer (NK) cells [9, 10]. Preclinical studies have also shown that the antitumor effects of IL-12 are most pronounced when given systemically [11]. Unfortunately, clinical use of recombinant IL-12 systemically has been complicated by inadvertent overstimulation in the form of systemic inflammatory response syndrome (SIRS) and T cell exhaustion (TCE) [12], as high loading doses of free protein were needed to ensure adequate distribution to target tissues. Nevertheless, while the side-effect profiles of systemic high-dose IL-12 administration are toxic, low doses of IL-12 are generally safe [13]. If formulated correctly, recombinant IL-12 may be used to alter the local cytokine environment and encourage antitumor immunity at a point far enough upstream in the inflammatory cascade to induce a multimodal downstream response, ultimately leading to a decreased likelihood of treatment resistance. Therefore, low-dose immunostimulatory cytokines coupled with proper real-time patient monitoring to ensure immune safety may produce subtle yet clinically beneficial antitumor immune activity without unwanted overstimulation [14].

Poly(lactide-co-glycolic) acid (PLGA) drug delivery vectors are Food and Drug Administration (FDA) approved and can elute a wide variety of substances as the polymer coating breaks down into metabolic intermediates [15]. Drug solubility, bioavailability, and particle stability can be individually altered by the organic coating, allowing for large shifts in the pharmacokinetic and pharmacodynamic properties of the encapsulate [16]. The negatively charged surfaces of PLGA particles are repelled by the glycocalyx which, along with their smaller size, allows for increased deposition within the interstitial space where they can elute their contents undisturbed [17]. Furthermore, to be used in systemic settings (versus intratumoral injections), nanospheres must be able to achieve safe and effective travel through the microvasculature of an organism (with capillaries being approximately 4-9 *μ*m in diameter) with minimal risk of forming emboli [18]. Encapsulating IL-12 within PLGA nanospheres is a potential strategy to achieve adequate biodistribution and tissue deposition of sensitive protein molecules without the need for toxic loading doses that resulted in the failure of clinical trials in the past [13]. While there have been several studies describing the synthesis of IL-12-loaded microspheres [19–35], to date, successful submicron encapsulation and elution of a structurally intact protein have not been well established. In this manuscript, we describe the synthesis and characterization of IL-12-loaded nanospheres (IL-12-NS), as well as the *in vivo* cytokinome profile produced when administered systemically.

## 2. Materials and Methods

### 2.1. Materials

Dichloromethane (DCM, #320269), Resomer RG 756 S (PLGA, #719927), NaCl (#7647-14-5), and poly(vinyl alcohol) (PVA, #341584) were purchased from Sigma-Aldrich (St. Louis, MO). Albumin from bovine serum (BSA), FITC conjugate (BSA-FITC, #A23015), penicillin-streptomycin 10,000 U/mL (Pen-Strep, #15140122), and Alexa Fluor 647 carboxylic acid, tris(triethylammonium) salt (Alexa 647, #A33084) were purchased from Thermo Fisher Scientific (Waltham, MA). Recombinant mouse IL-12 (p70) (carrier free) (rmIL-12, #577008) and mouse IL-12 (p70) ELISA MAX deluxe ELISA kits (#433606) were purchased from BioLegend (San Diego, CA). Gibco Fetal Bovine Serum Qualified Heat Inactivated US Origin (HI-FBS, #MT35011CV) and Corning Cell Culture Buffers: Dulbecco's Phosphate-Buffered Salt Solution 1X (DPBS, #21031CV) were purchased from Fisher Scientific (Pittsburgh, PA). Female BALB/c mice (6-8 weeks of age) (#000651) were purchased from the Jackson Laboratory (Bar Harbor, ME).

### 2.2. Synthesis of Blank and Alexa 647-, BSA-FITC-, and rmIL-12-Loaded PLGA Nanospheres Using the Double Emulsion/Solvent Evaporation (DESE) Method with Microsphere Removal and Ultracentrifugation

To create the oil phase, 800 mg of Resomer RG 756 S PLGA was dissolved in 32 mL DCM at room temperature (RT) for two hours using a magnetic stir bar at 500 RPM. To create the aqueous phase (2% PVA) of the emulsion, 2400 mg PVA and 96 mg NaCl were dissolved in 120 mL deionized water and microwaved for 10-second bursts in a standard kitchen microwave on the high setting until clear, then cooled on ice. Next, the first emulsion was made by suspending the encapsulation substrate (Alexa 647 [5 mg], BSA-FITC [5 mg], or rmIL-12 [25 *μ*g]) in 1200 *μ*L DPBS and adding to the oil phase, which was promptly stirred at 17500 RPM for 6 minutes on ice using a tissue homogenizer. Blank particles were prepared similarly, however, with no encapsulate. The second emulsion was formed by slowly pouring the first emulsion into 120 mL of the 2% PVA salt solution while being emulsified with the tissue homogenizer at 17500 RPM and continuing for a total of 8 minutes. The resulting suspension was then stirred for 16 hours with a magnetic stir bar at 750 RPM to evaporate the organic solvent. Once the solvent was evaporated, the resulting solution was spun at 3500 RPM thrice; following each spin, supernatant was collected and placed on ice, with the resulting pellet being resuspended. The particles were then washed twice with deionized water via ultracentrifugation at 20000 RPM for 40 minutes at 4 degrees Celsius before flash-freezing in liquid nitrogen and storing short term at -20 degrees Celsius.

### 2.3. Nanosphere Morphology

The morphology of the nanospheres was determined via scanning electron microscopy (SEM) using a Hitachi S-4700 scanning electron microscope (Tarrytown, NY). Briefly, lyophilized samples were mounted on metal stubs with carbon tape and prepared for imaging with a gold-targeting Denton Desk V sputter and carbon coater (Moorestown, NJ), which applies a thin layer of gold to the biosample under an argon gas atmosphere. To test the stabilizing ability of the sugar additive trehalose during the lyophilization process, 1 mL of 50 mmol/mL trehalose was added to a 1 mL aliquot of blank nanoparticles suspended in deionized water for a final trehalose concentration of 25 mmol/mL prior to lyophilization and subsequent gold sputter/SEM imaging.

### 2.4. Nanosphere Characterization

Nanosphere count and size distribution were determined in duplicate using the Malvern Panalytical NanoSight NS300 (Malvern, UK) at RT in deionized water with dilution factors of 1 : 50 and 1 : 14 for unloaded and rmIL-12-loaded batches, respectively. Nanosphere zeta potentials were determined using the Malvern Panalytical Zetasizer Nano Z at RT in deionized water with dilution factor of 1 : 50 for both unloaded and loaded batches. Results included are the product of biological duplicates (*n* = 2).

### 2.5. Nanosphere BSA-FITC Encapsulation

Z-stack images of BSA-FITC-loaded PLGA nanospheres were created using the Zeiss 710 confocal microscope (Cambridge, UK).

### 2.6. Nanosphere rmIL-12 Elution Profile

500 million particles/mL of IL-12-NS were prepared in a nanosphere release buffer (NRB, 10% HI-FBS and 100 units/mL Pen-Strep in DPBS). At specified time points, nanospheres were pelleted at 10000 × *g* for 15 minutes, and an aliquot of supernatant was sampled. In between sampling times, suspensions were incubated at 37 degrees Celsius with continuous agitation (750 RPM) using a Benchmark Scientific MultiTherm Cool-Heat-Shake (Edison, NJ). Each aliquot was stored at 4 degrees Celsius for at least 24 hours to equilibrate with the release buffer before determining rmIL-12 concentration through ELISA. Results included are the product of biological duplicates (*n* = 2).

### 2.7. Estimation of Encapsulation Efficiency (EE)

The amount of IL-12 encapsulated and released by the IL-12-NS was estimated by summing the protein concentrations measured by ELISA over time. This sum was multiplied by the particle concentration (PC) as determined by NanoSight and the total volume of synthesized particles (V); this value was then divided by the total mass of IL-12 added during synthesis (25 *μ*g) as shown in the following equation:

(1) $$\begin{array}{c} \text{EE}=\frac{\left(\sum_{i=0}^{i=5}\text{p}\text{gIL}‐12_{i}\right)*\text{PC}*V}{25\;\mu \text{g}}. \end{array}$$

Results included are the product of *n* = 2 biological duplicates.

### 2.8. *In Vivo* Alexa 647-Loaded PLGA Nanosphere Substrate Biodistribution and Safety Study

Female BALB/c mice received 1 mg/kg intravenous (tail vein) or intraperitoneal (i.p.) injections of Alexa 647-loaded PLGA nanospheres suspended in sterile saline. The In Vivo Imaging System (IVIS® SpectrumCT In Vivo Imaging System, PerkinElmer, Waltham, MA) was used to monitor fluorescence intensity and biodistribution over a 30-minute interval, at which time animals were humanely euthanized by CO_2_ asphyxiation and their femurs and lungs harvested for Z-stack confocal microscopy (Zeiss Violet Confocal, Jena, Germany).

### 2.9. *In Vivo* Administration of IL-12-Loaded PLGA Nanospheres and Cytokine Analysis

Thirty female BALB/c mice received retroorbital (r.o.) administration of 250 million IL-12-loaded nanospheres in 250 *μ*L sterile saline. Groups of 3 mice were euthanized at the following time points: 5 minutes, 6 hours, 12 hours, 24 hours, 48 hours, 72 hours, 96 hours, 11 days, 18 days, and 25 days (*n* = 3). At each time point, blood was collected through cardiac puncture. Blood concentrations of interferon-gamma (IFN-*γ*), IL-10, IL-12p70, IL-1*β*, IL-2, IL-4, IL-5, IL-6, chemokine (C-X-C motif) ligand 1 (CXCL-1), and tumor necrosis factor-alpha (TNF-*α*) were analyzed using the Meso Scale Discovery (Rockville, MD) V-PLEX Proinflammatory Panel 1 Mouse Kit per manufacturer protocol. Treated animals were compared to pooled control animal samples using Student's *t* test with *α* = 0.05.

## 3. Results

### 3.1. Nanosphere Synthesis, Morphology, and Characterization

Unloaded (blank), Alexa 647-, BSA-FITC-, and rmIL-12-loaded PLGA nanospheres (IL-12-NS) were successfully synthesized using the DESE method with ultracentrifugation as described. The morphology of both blank (Figures 1(a)–1(c)) and rmIL-12-loaded (Figures 2(b) and 2(c)) PLGA nanospheres was determined using scanning electron microscopy (SEM) to be spherical in shape with a mean particle diameter of 201.7 ± 6.7 nm and 138.1 ± 10.8 nm, respectively; the blank and rmIL-12-loaded PLGA nanosphere counts for each batch were determined to be 6.49 × 10^9^ ± 6.19 × 10^8^ particles/mL and 1.66 × 10^9^ ± 4.45 × 10^8^ particles/mL, respectively (Table 1). The introduction of 25 g rmIL-12 during particle synthesis resulted in a decrease in zeta potential magnitude from −21.3 ± 0.808 mV to −15.1 ± 1.249 mV (Table 1).

### 3.2. Nanosphere BSA-FITC Encapsulation and Z-Stack Imaging

To determine whether the synthesized nanospheres could indeed encapsulate protein and not merely adsorb it to the outer surface, 5 mg FITC-labeled BSA was loaded into the nanospheres; the resulting batch was imaged using confocal microscopy to visualize the internal structure. As shown in Figure 2(a), Z-stacking analysis confirmed that BSA was both adsorbed to the surface and incorporated within the polymeric shell.

### 3.3. IL-12-NS Elution Profile

500 million particles/mL of IL-12-NS were eluted in NRB; aliquots taken daily were subsequently analyzed with ELISA for heterodimeric p70 rmIL-12 concentrations released over time. The elution profiles for each particle concentration are shown in Figure 3, which displayed “burst” (days 0-1) and “sill” (days 1-5) phases characteristic of PLGA particle nanoencapsulation [36].

### 3.4. Estimation of Encapsulation Efficiency (EE)

The amount of encapsulated rmIL-12 available for elution was estimated using Equation (1), and EE was determined to be 0.101 ± 0.009% (Table 1).

### 3.5. *In Vivo* Alexa 647-Loaded PLGA Nanosphere Substrate Biodistribution and Safety

We sought next to investigate whether the contents of PLGA nanospheres distribute systemically following injection without adverse events, including death. To accomplish this goal, PLGA nanospheres were loaded with Alexa 647 and administered to female BALB/c mice either intravenously (via tail vein) or intraperitoneally (i.p.) and monitored through IVIS imaging. At 30 minutes postinjection, both routes of administration resulted in systemic distribution of nanosphere contents (Figure 4(a)) without any signs of morbidity or mortality. Fluorescent microscopy following necropsy showed distribution of the encapsulate to both the lung and bone (Figure 4(b)).

### 3.6. *In Vivo* Characterization of Cytokinome Profile Induced by the Administration of IL-12-NS

We next evaluated the *in vivo* cytokinome profile induced by intravenous injection of 250 million IL-12-NS into BALB/c mice. This concentration was chosen because it was the highest particle count: saline ratio the mice could tolerate retroorbitally (data not shown). Following injection, groups of three [3] mice were euthanized at a total of ten [10] time points over the course of 25 days and blood cytokine concentrations were determined, normalized to control mice, and presented as the fold change from physiological baseline. For reference, a fold change of one (1) indicates equal cytokine levels in comparison to control, whereas a fold change of two (2) or one-half (0.5) indicates a respective doubling or halving from physiological levels. Although an oversimplification, for charting purposes, the cytokines were split into three groups by their generalized tumor-destroying (IFN-*γ*, IL-2, and IL-5), tumor-promoting (IL-10 and IL-4), or SIRS-associated (IL-1*β*, IL-6, CXCL-1, and TNF-*α*) properties [37–62].

#### 3.6.1. Tumor-Destroying Cytokines: IFN-*γ*, IL-2, and IL-5

During the burst phase, blood concentrations of IFN-*γ* were significantly increased at 6 hours (*p* < 0.05) but significantly decreased at 12 hours (*p* < 0.05) (Figure 5(a)). During the sill phase, IFN-*γ* was also significantly decreased at 48 and 72 hours (*p* < 0.05); however, it showed a positive trend across the sill phase (*R* = 0.77), with IFN-*γ* being elevated an average of 3.08-folds over the control at 25 days postinjection (*p* = 0.052, Figure 5(b)).

IL-2, albeit below physiologic levels, showed no significant fold changes during the burst phase (Figure 5(a)) but was significantly decreased at day 18 (*p* < 0.05) (Figure 5(b)). Further, it showed a positive trend across the sill phase; however, it did not return to baseline production levels during the 25-day sampling period (*R* = 0.48, Figure 5(b)).

Much like IL-2, IL-5 showed no significant fold changes during the burst phase (Figure 5(a)) but was significantly decreased at 24 hours postinjection (*p* < 0.05) (Figure 5(b)). Similar to IFN-*γ*, IL-5 also showed a positive trend across the sill phase, exceeding physiological levels at both the 11- and 18-day time points postinjection although it was not statistically significant (Figure 5(b)).

#### 3.6.2. Tumor-Promoting Cytokines: IL-10 and IL-4

Tumor-promoting cytokines IL-10 and IL-4, though elevated in the 6-hour sample, showed no significant changes during the burst phase (Figure 5(c)). However, during the sill phase, IL-10 and IL-4 concentrations trended downward and remained near or below physiological levels after the 72- and 48-hour time points, respectively (*R* = −0.51 and −0.37, respectively, Figure 5(d)).

#### 3.6.3. SIRS-Associated Cytokines: IL-1*β*, IL-6, CXCL-1, and TNF-*α*

IL-1*β*was significantly increased at only the 6-hour time point (*p* < 0.05) throughout the 25-day sampling period postinjection during both the burst (Figure 5(e)) and sill phases (Figure 5(f)). It also showed a negative correlation across the sill phase, returning from those elevated levels to at or below physiological levels (*R* = −0.54, Figure 5(f)).

IL-6 was significantly elevated during the burst phase at 6- (*p* < 0.01) and 12- (*p* < 0.001) hour time points, reaching a transient maximum of a 30.58-fold increase over the control at 6 hours (Figure 5(e)). During the sill phase, IL-6 remained significantly increased at 24 hours (*p* < 0.05), 48 hours (*p* < 0.01), 96 hours (*p* < 0.001), and 18 days (*p* < 0.05) but, overall, trended downward (*R* = −0.60) and was statistically equivalent to the control by 25 days (Figure 5(f)).

During the burst phase, CXCL-1 was significantly elevated at 5 minutes (*p* < 0.05), 6 hours (*p* < 0.001), and 12 hours (*p* < 0.05). During the sill phase, it was significantly increased at 24 hours (*p* < 0.01) but displayed an overall negative correlation, returning to near baseline levels by the 72-hour time point (*R* = −0.60, Figure 5(f)).

TNF-*α* was significantly decreased during the burst phase at 5 minutes (*p* < 0.05) and 12 hours (*p* < 0.001) (Figure 5(e)). During the sill phase, TNF-*α* was significantly increased at 48 and 72 hours (*p* < 0.05) (Figure 5(f)). Interestingly, TNF-*α* was significantly decreased at 25 days (*p* < 0.01) (Figure 5(f)). Similar to the other SIRS-associated cytokines mentioned previously, TNF-*α* showed a negative correlation across the sill phase, returning to normal physiologic levels (*R* = −0.46, Figure 5(f)).

## 4. Discussion

Multiple cytokines have been shown to exhibit potent antitumor properties in preclinical studies; examples include IL-12, IL-2, IL-17, and IFN-*γ* among others [63]. IL-12, produced mainly by tumoricidal T_H_1 cells, showed promise in animal models against a wide variety of tumor types including sarcoma, with best responses achieved through systemic versus local (intratumoral) administration [11]. Unfortunately, recombinant IL-12 cytokine therapy thus far has produced underwhelming results in human patients. Clinical trials conducted in the 1990s required high loading doses of IL-12 to achieve adequate tissue biodistribution and resulted in TCE, SIRS, and ultimately worse outcomes [13]. In contrast, low-dose IL-12 given over prolonged periods has been shown to induce tumor regression without overstimulation, though there are currently few cases reported in the literature using this treatment strategy [64, 65]. Encapsulation in PLGA nanospheres may provide an opportunity to achieve slow and controlled delivery of IL-12 in a systemic fashion while ensuring delivery of contents to peripheral tissues.

IL-12-NS eluted picogram-scale protein doses corresponding to the equivalent of approximately 2-3.3 ng over the course of five days, and their diameter fell within a size distribution range of 100-200 nm. Notably, the zeta potential of loaded batches decreased in magnitude an average of 6.2 mV, which may reflect adsorption of rmIL-12 to the outer shell of the polymer coating [66]. The EE of our synthesis method was low (0.101%) and likely was due to the incorporation of rmIL-12 within microspheres, which comprises most of the formed product and is ultimately discarded during nanosphere purification. While other methods of synthesis (e.g., sonication) could have been employed for better encapsulation, bioactive IL-12 has a dimeric structure and is held together by a single disulfide bond that could easily be disrupted by vigorous agitation methods.

The *in vivo* studies provide a glimpse of the effects of IL-12-NS therapy on the systemic immune system. The biodistribution study suggested that the PLGA nanospheres (1) did not immediately flocculate and subsequently embolize and (2) distributed their contents systemically. As our group is primarily interested in metastatic osteosarcoma, we were especially excited to witness the distribution of nanosphere contents to the bone and lung. Further, V-PLEX analysis revealed significant changes in the cytokinome profiles of IL-12-NS-treated mice. Corresponding to the leukopenia observed in clinical trials following exogenous IL-12 administration, IFN-*γ* nadir occurred at 72 hours; however, in contrast to clinical trials, levels recovered quickly and displayed positive correlations postburst out to 25 days [67, 68]. The rapid recovery of secretory capacity following IL-12-NS administration suggests a lower likelihood of irreversible overstimulation.

Further, while serum IFN-*γ* levels in early clinical trials showed increasingly diminished responses to IL-12 over time, IL-12-NS-treated mice showed the opposite trend, which started at the onset of the sill phase and remained out to 25 days. Moreover, IL-12-NS administration induced these proinflammatory changes while prompting minimal counterregulatory increases in anti-inflammatory IL-10 and IL-4 cytokine levels [69, 70]. As SIRS is the most feared complication of recombinant cytokine therapy, IL-12-NS-induced increases in SIRS-associated cytokines could indicate dose-limiting toxicity. Although IL-6 levels increased to 30-folds of the baseline during the burst phase, they normalized by 72 hours and trended negatively throughout the sill phase. Similar trends were observed with IL-1*β* and CXCL-1, suggesting the potential for immune recovery and decreased likelihood of progression to a SIRS-like state. The increase of IFN-*γ* over time alongside the negative correlate of IL-10 and little to no change in TNF-*α* as well as IL-6 suggests that repeated administration of low-dose IL-12 through the vector system IL-12-NS may not produce an exhaustive cytokinome believed to be associated with treatment failures in previous clinical trials [71]. Given the initial increase in IFN-*γ* with a sustained increase over several weeks in conjunction with a short increase in TNF-*α* that normalizes quickly (within 96 hours), and IL-10 levels that essentially never change, the cytokinome is set perfectly to achieve sustained immunostimulation without firing the immunosuppressive response. All of these positive responses are seen despite utilizing logarithmically lower doses than those delivered during human clinical trials (even when calculated as a ng/kg/day dosing assessment). These data further suggest the importance of the vector system which safely creates the antitumor, immunostimulatory environment sought by previous researchers.

## 5. Conclusion

From these results, we conclude that rmIL-12 can be effectively packaged into PLGA nanospheres using the double emulsion/solvent evaporation (w1/o/w2) technique with ultracentrifugation and can achieve a homogenous distribution with a mean particle diameter of 138.1 ± 10.8 nm. Additionally, the nanospheres produced a characteristic elution profile with early “burst” and late steady-state “sill” phases with an average steady-state elution of 15 picograms IL-12/day at a starting concentration of 250 million spheres/mL. For the *in vivo* portion of the study, we found that IL-12-loaded nanospheres produced a systemic cytokine profile favoring immunostimulation without long-term elevation of SIRS-inducing acute phase response cytokines. While a larger experimental group may need to be tested to further validate our results, we suggest that IL-12-loaded nanospheres can produce antitumor immune profiles without inducing TCE and SIRS which is deserving of further investigation.

## Figures and Tables

**Figure 1:** Scanning electron microscopy (SEM) images of unloaded (blank) poly(lactide-co-glycolic) acid (PLGA) nanospheres lyophilized without (a, b) and with (c) 25 mM trehalose at 2500x, 9000x, and 5000x magnifications, respectively.

**Figure 2:** (a, b) Scanning electron microscopy (SEM) images of lyophilized recombinant mouse IL-12- (rmIL-12-) loaded PLGA nanospheres at 8000x and 25000x magnifications, respectively. (c) Fluorescein isothiocyanate- (FITC-) conjugated bovine serum albumin (BSA) was loaded into poly(lactide-co-glycolic) acid (PLGA) nanospheres, and the product was visualized for protein incorporation through confocal microscopy.

**Figure 3:** Cumulative amount of protein eluted over time from recombinant mouse IL-12-loaded poly(lactide-co-glycolic) acid (PLGA) nanospheres at a concentration of 500 million particles/mL as measured by ELISA. Nanospheres were eluted in 500 *μ*L of release buffer (NRB; 10% heat-inactivated fetal bovine serum [HI-FBS] and 100 units/mL Pen-Strep in DPBS) under constant agitation. Samples were collected from the supernatant following centrifugation of the pellet at 10000 × *g* for 15 minutes at 4 degrees Celsius.

**Figure 4:** Female BALB/c mice were inoculated with 1 mg/kg of Alexa 647-loaded nanospheres dissolved in sterile saline and monitored for fluorophore distribution (a) systemically over 30 minutes (images presented by time from top [initial tail vein injection], middle [initial i.p. injection], to bottom [30 minutes postinjection]) via IVIS imaging through i.p. (left) and tail vein (right) injections (∗ indicates IVIS signal immediately following either injection) and (b) in the bone (left) and lung (right) at four hours postinjection via fluorescent microscopy.

**Figure 5:** Blood cytokine concentrations of *n* = 3 mice euthanized at various time points following retroorbital inoculation of 250 million recombinant mouse IL-12-loaded PLGA nanospheres. Samples normalized to six control mouse cytokinomes and represented as fold change. For reference, a fold change of one (1) indicates equal cytokine levels in comparison to control, whereas a fold change of two (2) or one-half (0.5) indicates a respective doubling or halving from physiological levels. Tumor-destroying cytokines, IFN-*γ*, IL-2, and IL-5, were sampled at (a) the burst phase—5 minutes (5 m), 6 hours (6 h), and 12 hours (12 h), and (b) the sill phase—24 hours (24 h), 48 hours (48 h), 72 hours (72 h), 96 hours (96 h), 11 days (11 d), 18 days (18 d), and 25 days (25 d), postinoculation. Tumor-promoting, IL-10, IL-4, and IL-5 (c, d), and SIRS-associated, IL-1*β*, IL-6, CXCL-1, and TNF-*α* (e, f), cytokines are also displayed at the same time points, graphically separated into burst and sill phases. Statistical differences were determined using Student's *t* test. ^∗^*p* < 0.05, ^∗∗^*p* < 0.01, and ^∗∗∗^*p* < 0.001.

**Table 1:** 

	Average particle count (particles/mL)	Average *ζ* potential (mV)	Average EE (%)
Unloaded	6.49 × 10^9^ ± 6.19 × 10^8^	−21.3 ± 0.808	N/A
Loaded	1.66 × 10^9^ ± 4.45 × 10^8^	−15.1 ± 1.249	0.101 ± 0.009

EE: encapsulation efficiency (%).

## Data Availability

The datasets generated and/or analyzed in the current study are available from the corresponding author on reasonable request.
